The article "Determination of the Level of Heavy Metals in the Selected Cereals from Debre Markos Local Market, Amhara Region, Ethiopia" was published in 2022. Journal: Int J Anal Chem.

# Determination of the Level of Heavy Metals in the Selected Cereals from Debre Markos Local Market, Amhara Region, Ethiopia

**DOI:** 10.1155/2022/7146439

**Published:** 2022-12-05

**Authors:** Amsalu Getu, Yimer Seid, Biset Asrade

**Affiliations:** ^1^Department of Pharmacy, College of Medicine and Health Sciences, Wollo University, Dessie, Ethiopia; ^2^Metema District Hospital, Amhara Region, Metema, Ethiopia; ^3^Department of Pharmacy, College of Medicine and Health Sciences, Bahir Dar University, Bahir Dar, Ethiopia

## Abstract

**Background:**

Environmental contamination by heavy metals has become a worldwide problem in recent years because of industrial and agricultural development which causes cereal crop contamination via their wastes. The presence of toxic heavy metals in cereal crops accumulate in the body for a prolonged period of time which poses acute and chronic health risks. The aim of the study was to assess the level of heavy metals in selected cereals sold at Debre Markos local market, in Ethiopia.

**Methods:**

The samples were prepared for analysis by using the dry ashing method, and their cadmium, lead, chromium, and copper contents were analyzed by using microwave-induced plasma-atomic emission spectroscopy (MP-AES) and were expressed in mgkg^−1^ dry weight. The accuracy of the method was analyzed by the spike recovery test.

**Results:**

The percentage recovery for Cr, Cu, Pb, and Cd in each sample ranged from 85.6 to 112.8%. The levels of heavy metals (mean ± SD) were as follows: chromium, 2.20 ± 0.072, 2.22 ± 0.061, 1.57 ± 0.48, and 1.84 ± 0.26; copper, 2.94 ± 0.19, 2.31 ± 0.06, 1.28 ± 0.13, 1.52 ± 0.035, and 2.31 ± 0.06; lead, 0.49 ± 0.031, 0.34 ± 0.121, 0.52 ± 0.029, and 0.37 ± 0.15; and cadmium, 2.01 ± 1.73, 1.84 ± 1.60, 1.95 ± 1.69, and 1.93 ± 1.67 for barley, teff, wheat, and maize, respectively. This study revealed that the levels of Cr and Cu are generally below the permissible limit. However, the levels of Pb and Cd in all cereal samples were found to be above the permissible limit set by FAO/WHO, 0.2 and 0.1 mg kg^−1^, respectively.

**Conclusion:**

The findings of the study suggest that most of the analyzed crops contained unsafe levels of lead and cadmium that exceeded the WHO permissible limits. Therefore, regular monitoring of these toxic metals in cereal crops should be carried out to prevent heavy metal toxicity associated with the consumption of some cereal crops marketed in the Debre Markos local market, Ethiopia.

## 1. Introduction

Environmental contamination by heavy metals has become a worldwide problem in recent years due to the fact that heavy metals are not biodegradable [1], have a long biological half-life, and can be bio-accumulated through the biological chain [2]. Heavy metals are among the major contaminants of food and may be a major problem to the environment. Heavy metals may enter the human body through the consumption of contaminated drinking water, cereals and vegetables grown in metal-contaminated soil, industrial liquid waste, and sediments [1, 2]. Heavy metals are potential environmental contaminants that cause human health problems if present in a higher percentage in food grains, which indicates that food quality and safety have become a major public concern worldwide [3].

The article "Determination of the Level of Heavy Metals in the Selected Cereals from Debre Markos Local Market, Amhara Region, Ethiopia" was published in 2022. Journal: Int J Anal Chem.

Metals such as copper (Cu) and chromium (Cr-III) are essential nutrients that are required for various biochemical and physiological functions. But an inadequate supply of these micronutrients results in a variety of deficiency diseases or syndromes [4]. However, several hazardous heavy metals such as Pb, Cd, and Cr (VI) are classified as nonessential to metabolic and other biological functions [5, 6]. These metals are deleterious in various respects, and they have therefore been included in the top 20 list of dangerous substances by the United States Environmental Protection Agency and the Agency for Toxic Substances and Disease Registry [5, 6]. The strength of a toxic effect of all trace metals depends principally on the absorption, concentration, and persistence of the eventual toxicant at its location of action [7].

It is evident that prolonged consumption of foodstuffs with unsafe concentrations of heavy metals may lead to chronic accumulation of heavy metals in the kidney and liver of human beings, causing various disorders in numerous biochemical processes [8, 9]. Many of the toxic metals such as cadmium, lead, and chromium (VI) are carcinogens and are involved in various communicable and noncommunicable diseases (Alzheimer's disease, Parkinson's disease, osteoporosis, developmental disorders, and failure of several organs such as the heart, kidney, lungs, and immune system) [10, 11] due to which metal analysis in food is an essential aspect of food quality control [12, 13].

Agriculture is the mainstay of farmers in the study area but agricultural land degradation is one of the major problems in this area and leads to the depletion of natural organic matter which affects soil fertility and yields of crop production. So, to maintain the fertility of farmlands and to increase crop production, farmers frequently use modern practices such as compost (59.23%) and chemical fertilizers (diammonium phosphate and urea) (98.46%), and they also use other chemicals (pesticides and herbicides) which are the major source of heavy metals and are considered the most important health concern [14]. Recent studies conducted in different countries have shown contaminations of different foodstuffs particularly cereal crops contaminated with heavy metals such as cadmium, chromium, copper, and lead. However, in Ethiopia, there are no regulations and in-depth investigations of heavy metal accumulations in cereal crops and other foodstuffs particularly in the study area [1–7].

The article "Determination of the Level of Heavy Metals in the Selected Cereals from Debre Markos Local Market, Amhara Region, Ethiopia" was published in 2022. Journal: Int J Anal Chem.

Therefore, the major significance of the study is to provide concrete information about the level of heavy metals and health risk implications for the population consuming cereal crops cultivated in agricultural farmlands. It also gives a clue for further studies on the soil in the study area and cereals cultivated in different parts of the region. Furthermore, the outcome of this study will be more beneficial by creating awareness not only to consumers but also to agricultural institutions about the toxic effects of heavy metals.

## 2. Materials and Methods

### 2.1. Materials

#### 2.1.1. Equipment and Apparatus

A microwave-induced plasma-atomic emission spectroscope (Agilent 4210, MP-AES, USA), digital analytical balance (Mettler Toledo, Me204, Switzerland), vortex mixer (Mfr. S1-p236, USA), polyethylene bag, hot plate (digital hotplate, thermo-scientific, USA), vacuum oven (Digit heat, J. P. Selecta, Spain), Whatman filter paper (Man™, No. 41, UK), muffle furnace (saturate scientific, Great Britain), porcelain crucibles, electronic blender with stainless steel blades, mortar and pestle, and sieve (Retsch®, stainless steel, 850 *μ*m, Germany) were used for the determination of heavy metals in the cereal samples.

#### 2.1.2. Chemicals and Reagents

All chemicals and reagents used throughout the experiments were of analytical grade. Standard reference metals of chromium (Cr), copper (Cu), lead (Pb), and cadmium (Cd) of the 1000 ppm stock solution (BDH chemicals Ltd., Merck, England) were obtained from Ethiopian Public Health Institution (EPHI), Addis Ababa, Ethiopia. The solvents and chemicals used in this research experiment were ultrapure water (Milli-Q™ Water system, Darmstadt, Germany), HCl (37%, Sigma Aldrich, Sp. Gravity 1.19, USA), and HNO_3_ (70%, Sigma Aldrich, Sp. Gravity 1.4, USA).

### 2.2. Methods

#### 2.2.1. The Study Area and Period

The study was conducted at Debre Markos local market from October 2019 to August 2020. Debre Markos is the capital city of the East Gojjam zone, Amhara region, Northwest Ethiopia, and it is located 254 kilometers from Bahir Dar, the capital city of the Amhara region, and 305 kilometers from Addis Ababa, the capital city of Ethiopia (Figure 1). The city has a latitude and longitude of 10° 20′N 37° 43′E and an elevation of 2446 meters above sea level. The annual temperature and rainfall of the city are 15.9°C and 1321 mm, respectively. According to the 2007 census conducted by the Central Statistical Agency of Ethiopia, the East Gojjam zone has a total population of 2,153,937 [14], which is an increase of 26.68% over the 1994 census, of whom 1,066,716 are men and 1,087,221 women with an area of 14,004.47 square kilometers. There are 18 districts in the East Gojjam zone of Amhara National Regional State [14].

The article "Determination of the Level of Heavy Metals in the Selected Cereals from Debre Markos Local Market, Amhara Region, Ethiopia" was published in 2022. Journal: Int J Anal Chem.

#### 2.2.2. Sample Collection

The representatives of four cereal samples of barley, teff, wheat, and maize (Table 1, Figure 2) were collected randomly at Debre Markos local market from February 1 to February 28, 2020, during the harvest time. About one kg sample of each type of cereal was purchased randomly from 40 merchants (40 kgs total, 10 kgs each) within the market area available during the sample collection period and the samples were well mixed in a wide and flat tray to get about 10 kg of one bulk sample from each sample. From the total sample (10 kg), the subsample (1 kg, each) was considered quite representative for each type of cereal sample and was stored in polyethylene bags and brought to the laboratory for analysis [15, 16].

#### 2.2.3. Sample Digestion and Analysis

Analytical samples, 1 kg, were taken randomly from the composite samples and grounded directly by using an electric blending device. Then, the powder was passed through a 0.850 mm sieve and 5 g of grounded and homogenized powder samples were weighed and transferred to acid-washed porcelain crucibles which were labeled according to the type of the sample. The samples were heated on a hot plate at 110°C for 30 minutes under a hood to remove moisture and to dry the samples. The dried sample was transferred to a muffle furnace and the dry ashing method was carried out in the muffle furnace at 350°C until the samples were charred and then carrying out a stepwise increase of the temperature up to 550°C for two hours. One ml of water for wetting and 2 ml of concentrated nitric acid (HNO_3_) were added to the ash and it was evaporated to dryness on a hot plate under the hood and then placed and heated again in a muffle furnace to oxidize and destruct the remaining organic matter. The samples were left to ash for 30 minutes at 550°C and then the crucibles were cooled in a desiccator. After ashing was completed, the obtained product was dissolved in 5 ml of 6M HCl and digested on a hot plate to dryness for 30 minutes until white fumes ceased and the solution was colorless [17]. After cooling, the solution was filtered by using the Whatman filter paper No. 41 into a 50 ml standard volumetric flask and was diluted to the mark of 50 ml. Finally, the concentration of Pb, Cd, Cr, and Cu in each sample was determined using microwave plasma-atomic emission spectroscope obtained from the Ethiopian Public Health Institution (EPHI) (Addis Ababa, Ethiopia). Blank solution containing the only mixture of concentrated HNO_3_ and HCl was also prepared following the same digestion procedure used for the samples and was diluted up to 50 mL with deionized water. All experiments were carried out in triplicates.

The article "Determination of the Level of Heavy Metals in the Selected Cereals from Debre Markos Local Market, Amhara Region, Ethiopia" was published in 2022. Journal: Int J Anal Chem.

#### 2.2.4. Calibration Curve Procedure

Intermediate standard solution of 100 ppm was prepared from the standard reference stock solution of 1000 ppm of each metal by diluting 10 ml of standard reference metal with ultrapure water to a 100 ml solution to produce 100 ppm. From these intermediate stock solutions (100 mg/L), five working standard solutions (1 ppm, 5 ppm, 10 ppm, 15 ppm, and 20 ppm) of each metal were prepared for the calibration curve. The blank solution was prepared in parallel with the standard solution. Finally, the calibration curve was constructed using five-point calibration via the standard concentrations of the metals against the emission intensity of each metal.

#### 2.2.5. Determinations of Heavy Metals

The digested sample was analyzed to determine the concentration of Cr, Cu, Pb, and Cd by microwave plasma-atomic emission spectroscopy. Based on the average values of the three replicates, the concentrations of each heavy metal in the sample were determined from the calibration curve and the final concentration of heavy metals in 5 g of each sample in terms of mg/kg was determined using the following equation [1]:

(1) $$\begin{array}{c} Concentration\;in\;dr\;y\;weight\left(\frac{mg}{kg}\right)=\frac{C\left(mg/L\right)\times V\left(L\right)}{W\;}\text{,} \end{array}$$

where *C* (mg/L) is the concentration of the samples obtained from the calibration curve, *V* is the final volume (50 mL), and *W* is the initial weight (5 g) taken for sample analysis.

#### 2.2.6. The Recovery Test

A recovery study of the analytical procedure was carried out by spiking a known amount of the standard solution (1.25 mL of each standard heavy metal) of cereal samples (5 g for each sample), and the spiked samples were processed for analysis by using the dry ashing method as the same procedure used for unspiked samples. The percentage recoveries of the samples were calculated to evaluate the accuracy of the analytical procedure. Percent recovery was calculated by using the following equation [2]:

(2) $$\begin{array}{c} Percent\;Recovery\left(\%\right)=\frac{Concentration\;in\;spiked\;sample-concentration\;in\;un\;spiked\;sample}{actual\;concentration\;add\;e\;d\;}\times 100\text{.} \end{array}$$

The article "Determination of the Level of Heavy Metals in the Selected Cereals from Debre Markos Local Market, Amhara Region, Ethiopia" was published in 2022. Journal: Int J Anal Chem.

#### 2.2.7. Data Analysis

All quality control measures were taken including calibration check measures, determination of recovery test, and replicate analysis of the samples. The data were analyzed using SPSS version 23. The results were expressed as mean ± standard deviation (mg/kg dry weight) of triplicate analysis.

## 3. Results and Discussion

### 3.1. Accuracy and Precision

Percent recovery results of heavy metals ranged from 85.6 to 112.8% in the barley, teff, wheat, and maize samples (Table 2), and the values were within the acceptance range of 80 to 120% for metal analysis [17, 18], and also the percentage relative standard deviation (%RSD) values for all metals in a spiked sample was below 5% which was under the required control limits (≤10%) [19]. This indicates that the proposed analytical method is accurate and precise for the analysis of heavy metals. Therefore, the results obtained by this method are reliable, accurate, and precise. The correlation coefficient (*R*^2^) for Cr, Cu, Pb, and Cd ranged from 0.9966 to 0.9983 which was greater than the acceptance limit of the standards (≥0.995) [20], which indicates that there is a good correlation between heavy metal concentration and atomic emission intensity of each heavy metals in the specified concentration range (Table 2, Figures 3–6) [20].

### 3.2. Heavy Metal Concentrations in the Cereal Samples

The mean levels of Cr, Cu, Pb, and Cd in the selected cereal samples collected from the study area are given as the mean ± standard deviation (mg/kg) in dry weight and were determined using equation (1) after establishing linear regression equations (Table 2, Figures 3–6) by using the standard solutions of a triplicate digestion and triplicate analysis and presented in Table 3. The observed concentrations of Cr, Cu, Pb, and Cd in the cereals were compared with the recommended limit established by the FAO/WHO to assess the levels of its contamination [21].

Chromium was detected in all examined cereal samples and its values ranged from 1.57 mg/kg to 2.22 mg/kg. The mean levels of Cr were as follows: 2.20, 2.22, 1.57, and 1.84 mg/kg for barley, teff, wheat, and maize, respectively (Table 3), which is lower than the FAO/WHO permissible limit, 2.3 mg/kg, but the level of Cr in barley and teff was in the baseline of the FAO/WHO limit. It may pose a health risk to consumers due to gradual accumulation in the body through the consumption of these cereals as food products [21].

Copper was detected in all cereal samples and its values ranged from 1.28 to 2.94 mg/kg. The mean levels of copper were as follows: 2.94, 2.31, 1.28, and 1.52 mg/kg for barley, teff, wheat, and maize, respectively (Table 3), which is lower than the FAO/WHO permissible limit, 30 mg/kg. This result also showed that the copper level in the barley sample was higher than in the other cereal samples [21].

The article "Determination of the Level of Heavy Metals in the Selected Cereals from Debre Markos Local Market, Amhara Region, Ethiopia" was published in 2022. Journal: Int J Anal Chem.

Lead was detected in all cereal samples and its values ranged from 0.34 to 0.52 mg kg^**−1**^. The levels of lead in the study were as follows: 0.49, 0.34, 0.52, and 0.37 mg/kg for barley, teff, wheat, and maize, respectively (Table 3). The mean levels of lead in this study were above the FAO/WHO permissible limit, 0.2 mg kg^−1^. Hence, cereals are not safe for human consumption. It may cause problems such as brain damage, seizures, CNS disorders, kidney disease, GI disturbances, slight liver impairment, and damage to a child's central nervous system and reproductive system [21].

Cadmium was detected in all cereal samples and its value ranged from 1.84 to 2.01 mg kg^−1^. The mean levels of Cd in the samples were 2.10, 1.84, 1.95, and 1.93 mg/kg for barley, teff, wheat, and maize, respectively, as shown in Table 3. The results obtained in this study were higher than the permissible limit set by the FAO/WHO, 0.1 mg/kg for cereal grains and 0.2 mg/kg for wheat grains. So, consumers of cereals are likely to encounter health risks because the cereals are not safe for human consumption due to high Cd levels [21].

## 4. Conclusion

In this study, selected cereal samples collected from Debre Markos local market were analyzed for the heavy metal (Cr, Cu, Pb, and Cd) content, and the results revealed that most of the analyzed crops contained unsafe levels of lead and cadmium that exceeded the FAO/WHO permissible limits. Therefore, regular monitoring of these toxic metals in cereal crops should be carried out to prevent heavy metal toxicity associated with the consumption of some cereal crops marketed in Debre Markos local market, Ethiopia.

## Figures and Tables

**Figure 1:** Location of the study area.

**Figure 2:** List of crops commonly used by the community of Debre Markos town, Northwest Ethiopia.

**Figure 3:** Standard calibration curve for chromium.

**Figure 4:** Standard calibration curve for copper.

**Figure 5:** Standard calibration curve for lead.

**Figure 6:** Standard calibration curve for cadmium.

**Table 1:** List of crops commonly used by the community of Debre Markos town, Northwest Ethiopia.

S. No.	Common name	Scientific name
1	Barley	*Hordeum vulgare* L.
2	Teff	*Eragrostis tef* L.
3	Wheat	*Triticum aestivum* L.
4	Maize	*Zea mays* L.

**Table 2:** Recovery test results and calibration curve equations for the determination of heavy metals in selected cereals.

Analyte	Recovery (%)	Regression equations (*Y* = *mx* + *b*)^*∗*^	*R * ^2^	Wavelength (nm)
Cr	85.6–107.2	*Y* = 13969*x* + 3289.8	0.9973	425.433
Cu	91.6–106.4	*Y* = 103051*x* + 34163	0.9966	324.754
Pb	98.4–112.8	*Y* = 1899.4*x* + 200.23	0.9976	405.754
Cd	99.2–110.4	*Y* = 13829*x* + 4869.5	0.9983	228.802

^*∗*^ *Y* = intensity; *m* = slope; *x* = concentration (mg/L); *b* = intercept.

The article "Determination of the Level of Heavy Metals in the Selected Cereals from Debre Markos Local Market, Amhara Region, Ethiopia" was published in 2022. Journal: Int J Anal Chem.

**Table 3:** Average levels of heavy metals (mean ± SD, mg kg^−1^, dry weight) in the cereal samples.

Metals	Cereal samples				FAO/WHO limit (mg/kg)^a^
	Barley	Teff	Wheat	Maize
Cr	2.20 ± 0.072	2.22 ± 0.061	1.57 ± 0.48	1.84 ± 0.26	2.3
Cu	2.94 ± 0.19	2.31 ± 0.06	1.28 ± 0.13	1.52 ± 0.035	30
Pb	0.49 ± 0.301	0.34 ± 0.12	0.52 ± 0.029	0.37 ± 0.15	0.2
Cd	2.01 ± 1.73	1.84 ± 1.60	1.95 ± 1.68	1.93 ± 1.67	0.1

Source: ^a^FAO/WHO report, 2011.

## Data Availability

The data used to support the findings of this study are available from the corresponding author upon request.
